# The Effect of Individual Nursing on Anxiety and Depression in Patients with Temporomandibular Disorders

**DOI:** 10.1155/2022/7748696

**Published:** 2022-07-12

**Authors:** XiaoQiu Ke, Xia Shao, Jie Wang, JinFeng Zhuo

**Affiliations:** ^1^Department of Oral and Maxillofacial, The First Affiliated Hospital of Wenzhou Medical University, Wenzhou, Zhejiang, China; ^2^Department of Endocrinology, Yanbian University Hospital, Yanji, Jilin, China

## Abstract

**Objective:**

This study aimed to explore the effects of individualized nursing in patients with temporomandibular disorders (TMD).

**Methods:**

From June 2019 to April 2021, 80 patients with TMD were admitted to the First Affiliated Hospital of Wenzhou Medical University. Among them, 40 patients (control group, CG) received routine nursing and 40 patients (experimental group, EG) received individualized nursing. Functional exercise compliance, pain score, maximum mouth opening, nursing satisfaction questionnaire, self-rating anxiety scale, and self-rating depression scale were investigated.

**Results:**

From June 2019 to April 2021, 81 patients with TMD were admitted to the First Affiliated Hospital of Wenzhou Medical University. Among them, 40 patients (control group) received routine care and 41 patients (experimental group) received individual care. There were no significant differences in mouth opening and pain score between the two groups before surgery (*P* > 0.05), but there were significant differences in mouth opening and pain score between the two groups 3 weeks after surgery. Patients' anxiety and depression were assessed by the SAS and SDS scores. Before nursing, the control group and experimental group (*P* < 0.05) had no significant difference. After nursing, the score of both groups decreased (*P* < 0.05). However, the score was lower in the experimental group, compared to the control group (*P* < 0.01).

**Conclusion:**

In summary, individualized nursing can improve patients' physical condition and reduce negative emotions and complications. In light of this, the study needs further verification by a large sample randomized controlled trial.

## 1. Introduction

Temporomandibular disorders (TMDs), one of the most prevalent diseases in the oral and maxillofacial region, is listed as the fourth oral-related disease affecting human health by the World Health Organization (WHO) for its large-scale multiple and outstanding refractory characteristics [1, 2]. The prevalence rate is 28.88%, with females more commonly affected than males [3, 4]. This disease usually originates from the temporomandibular joint (TMJ) on one side and compensatory overuse and movement of the contralateral TMJ due to unilateral chronic pain or motor impairment, some of which may gradually involve both sides [5]. Common causes include emotional stress, trauma, joint overload, and genetics. Due to frequent joint movement, the disease has a long treatment course, ranging from a few weeks to several years, and is also prone to recurrence [6]. Its pathogenesis is complex, and surgical treatment is required for patients who fail to receive conservative treatment [7]. The active degree of functional exercise in TMD patients receiving surgical treatment, in accordance with medical advice after discharge, directly affects postoperative rehabilitation and quality of life. However, due to patients' lack of understanding of the disease, the deficit in medical staff guidance, subjective conditions, and other factors, this results in low compliance of postoperative functional exercise with the progression of medical conditions. It is recognized that inpatients have more and more high requirements for medical services, and traditional nursing methods have been unable to meet the needs of all patients [8, 9].

Individualized nursing is a new nursing model developed on the basis of holistic nursing, which mainly embodies the higher realm of humanistic nursing and deepens the connotation of holistic nursing [10–12]. The individualized nursing intervention takes corresponding nursing and management measures according to each patient's clinical condition and psychological characteristics, improves the patient's comfort, moderation, and compliance, and helps the patient recover early and steadily [13]. The individualized nursing intervention is patient-centered, respects the individual differences of patients, and satisfies the reasonable needs of patients to the greatest extent. Moreover, psychological intervention can stabilize the patient's psychology and establish confidence by giving patients pain nursing intervention through medication, transfer of attention, and other methods to effectively control pain. Providing patients with diet nursing intervention, eating more food rich in vitamins, cellulose, and high protein can improve the recovery of gastrointestinal function [14]. Furthermore, the incidence of complications can be reduced, and the length of hospital stay can be shortened by nursing patients' complications, preventing postoperative infection, regularly assisting turning over, and assisting sputum discharge by tapping on the back. In previous studies [15–18], the application of individualized nursing in cancer and acute myocardial infarction was introduced, but the application effect of this method in patients with TMD was not used. Herein, in this research, we aimed to individualize nursing carried out for TMD and to evaluate the effect of this nursing on patients' rehabilitation.

## 2. Materials and Methods

### 2.1. Study Population

This study was approved by the Ethics Committee of the First Affiliated Hospital of Wenzhou Medical University. Patients and their families were informed, willing to participate in the study, and signed informed consent forms.

Patients with TMD admitted to the First Affiliated Hospital of Wenzhou Medical University from June 2019 to April 2021 were investigated. Inclusion criteria were as follows: (1) patients were diagnosed with TMD, and the diagnosis was confirmed by a stomatologist; (2) above 18 years old; (3) clear consciousness, normal mental state, ability to accurately express their own will, understanding the scoring scale, and cooperating with treatment; (4) the course of the disease is more than 3 months.

Exclusion criteria were as follows: (1) patients with severe systemic diseases and their complications, serious infections, and major diseases of viscera, tissues, and systems; (2) patients suffering from mental diseases; (3) patients not cooperating with treatment or poor compliance. The occurrence of any of the above is in accordance with the exclusion criteria.

### 2.2. Nursing Methods

Patients are free to choose on admission. Patients in both groups were given routine nursing. If there was any variation, the attending doctor was timely informed, and symptomatic treatment was given according to the doctor's advice. The nursing staff kept the sheets clean and tidy and regularly sterilized and ventilated the ward. They advised patients with TMD to eat a light and easily digestible diet. The experimental group was given individualized nursing. Nursing workers with robust theoretical knowledge and rich work experience led the discussion according to the patient's condition and determined the corresponding nursing intervention mode. (1) Pretreatment nursing intervention: nursing staff closely observed patients' psychological and mental state and provided psychological comfort and guidance for patients' individual psychological state. Understanding the patient's condition in detail: the patient's condition was discussed with the patient, the latter was encouraged to communicate with a recovering patient with the same similar diagnosis, the patient's confidence was enhanced, and the treatment compliance was improved. (2) Nursing intervention treatment: nursing staff encouraged patients and relieved their emotions during treatment to keep them relaxed. Attention was paid to the patient's facial condition, vital signs, and other indicators during the operation. After treatment, patients were assisted in recovering to a comfortable sitting position, and the body tension was relaxed. The patient was further instructed to take antibiotics to prevent infection. (3) Post-treatment nursing intervention: the diet of patients was guided, a reasonable collocation of nutrition supply was ensured, and disease recovery was promoted. The complete treatment plan and the advantages were discussed with the patient, the method of self-psychological adjustment was provided, and the patient was encouraged to eliminate the disease to the patient's psychological pressure. Nursing staff actively communicated with patients and their families to eliminate strangeness, and family members were advised to provide emotional support and solve emotional problems. Furthermore, disease knowledge to patients was popularized, and causes, treatment measures, precautions, and adverse reactions were clarified. Patients' questions were answered, and their emotional changes were observed. Patients were encouraged to read books, watch movies and television, and listen to music as a distraction. During the treatment, nurses were required to inform patients of the main points and matters needing attention in the treatment process. (4) Ward care: the number of ward visits was increased to 3 times a day, and patients' vital signs were closely monitored; the influence of noise and bright light were avoided to ensure an adequate resting environment and improve comfort and sleep quality.

### 2.3. Observation Indexes

(1) Maximum mouth opening (MMO): the vertical distance between the upper and lower central incisors at the maximum opening of the patient. The maximum mouth opening of the 2 groups was measured before surgery and 3 weeks after surgery. (2) Pain score: visual analog scale (VAS) was employed to evaluate the pain degree of patients in the two groups by 1∼10 points before surgery and 3 weeks after surgery. (3) Negative emotions: self-rated anxiety scale (SAS) and self-rated depression scale (SDS) were used to evaluate patients' negative emotions. They included 20 symptoms and assessed the frequency of symptoms. A score below 50 was considered normal, a score of 50–60 was considered mild, a score of 61–70 was considered moderate, and a score of over 70 was deemed severe. The higher the score, the more severe the symptoms in that area.

### 2.4. Statistical Methods

Continuous variables are presented as the mean + standard deviation (SD), and the *t*-test was used for comparison. Categorical data are summarized as frequencies or percentages. We used the chi-square to determine significant differences among the study groups. The data were analyzed by the R software version 4.00 (https://www.r-project.org/). *P* < 0.05 was considered statistically significant.

## 3. Results

### 3.1. General Information

From June 2019 to April 2021, 81 patients with TMD were admitted to the First Affiliated Hospital of Wenzhou Medical University. Among them, 40 patients (control group) received routine care, and 41 patients (experimental group) received individual care. General data for patients are shown in Table 1. No significant differences were observed in baseline data such as sex, age, and BMI (*P* > 0.05).

### 3.2. Maximum Mouth Opening and Pain Score

There were no significant differences in mouth opening and pain score between the two groups before surgery (*P* > 0.05), but there were significant differences in mouth opening and pain score between the two groups 3 weeks after surgery (*P* < 0.05).  Table 2 shows the results in a tabular format.

### 3.3. Emotional Scores of Patients in Control Group and Experimental Group

Patients' anxiety and depression were assessed by the SAS and SDS scores.  Table 3 shows the results in a tabular format. Before nursing, the control group and experimental group (*P* < 0.05) had no significant difference. After nursing, the score of both groups decreased (*P* < 0.05). However, the score was lower in the experimental group, compared to the control group (*P* < 0.01).

## 4. Discussion

Surgery is usually indicated for the clinical treatment of TMD [19], and its efficacy is not ideal. In order to promote the early recovery of patients, we should take targeted nursing measures according to the actual situation of patients. In this study, we provided individualized nursing to patients with TMD. The results reveal that individual nursing can enhance and promote patients' joint function recovery and nursing satisfaction, and reduce the occurrence of negative emotions [20, 21]. This demonstrates that the individual nursing model is effective in promoting patient rehabilitation.

Traditional nursing in clinical practice is passive and usually performed after complications or adverse reactions [22]. The core theme of personalized nursing is people-oriented, reflecting humanistic care, actively developing professional and targeted nursing for patients, and offsetting the passive nursing model [23]. We required the nursing staff to formulate a scientific and reasonable nursing plan before implementing nursing interventions to have a clear understanding of the nursing content according to the patient's condition, needs, and disease risk assessment [24]. Patients with TMD lack awareness of the disease, and its complications may bring negative emotions such as anxiety and depression [25–27]. Psychological counseling for patients showed that individualized nursing could improve patients' anxiety and depression. Therefore, through active communication with patients, proper psychological counseling can not only enhance patients' understanding of the disease but also encourage patients to cooperate with the treatment actively. Therefore, it is essential to use appropriate and effective nursing measures to improve patients' bad moods to ensure smooth operation and facilitate subsequent recovery [28].

In this study, implying that individual nursing care can further improve negative moods in patients receiving TMD treatment [29, 30]. Numerous factors affect the postoperative negative psychology of patients receiving TMD treatment [31], among which preoperative fear of surgical risk, postoperative fear of incomplete recovery, difficulty in swallowing and drinking after an operation, and other factors will affect patients' psychology. Long-term negative emotions will not only affect the normal metabolism of the body but can also induce the body to produce a stress response, which is not conducive to surgery and postoperative rehabilitation. Patients with preoperative psychological counseling significantly eased worries about operation risks. Through psychological consultation, patients mastered the skills of self-regulating their moods and actively improving their bad moods, making patients face surgery with the best attitude. In addition, high-quality care takes patients at the center of the nursing model and combines advanced nursing concepts. From the patients' point of view, comprehensive nursing intervention is carried out from the aspects of the body, psychology, oral hygiene, daily life, and diet, and adequate preparation is made. Therefore, it can eliminate or reduce the negative emotions of patients [32].

In this study, the pain score and maximum mouth opening of patients in the 2 groups were determined. No significant difference was noted. The postoperative pain score of the experimental group was significantly lower than that of the control group. However, the maximum mouth opening of the experimental group was significantly greater than that of the control group. This observation reveals that individualized care can effectively promote recovery of postoperative joint function in TMD patients. The postoperative functional exercise aims to help the temporomandibular joint structure, and masticatory muscles adapt to the new range of motion, promote tissue healing, strengthen masticatory muscle strength, and improve the patient's language. Nausea and vomiting, traction of the wound, accidental swallowing or inhalation, and wound shedding are common complications of TMD. In our study, the overall incidence of complications was significantly reduced, while the study group reported significantly higher nursing satisfaction compared to the control group. This suggests that individual nursing can effectively reduce complications and improve the satisfaction of TMD patients.

Although our study shows that individualized care has favorable outcomes for TMD patients, there are some limitations. This study was limited by the relatively small sample size. Another limitation of our study was that the latter was a single-center study. Thus, the influence of individual nursing on patients' long-term psychological state after surgery still needs to be confirmed through multicenter studies with a large sample size in the future.

## Figures and Tables

**Table 1:** Comparison of general information between the two groups.

Characteristics	Control group	Experimental group	*P* value
*N*	40	41	

Age, years	24.6 ± 3.0	25.5 ± 3.3	0.210

Sex, *n* (%)			0.610
Female	29 (72.5%)	30 (73.2%)	
Male	11 (27.5%)	11 (26.8%)	

BMI	20.3 ± 3.5	19.9 ± 3.1	0.946

**Table 2:** Comparison of maximum mouth opening and pain score of two groups.

	Control group	Experimental group	*P* value
Maximum mouth opening			
Preoperation	31.0 ± 6.9	30.9 ± 6.3	0.740
3 weeks	28.2 ± 4.6	25.1 ± 4.3	0.002

Visual analog scale score			
Preoperation	6.7 ± 1.0	7.1 ± 1.1	0.179
3 weeks	3.3 ± 0.6	2.0 ± 0.7	<0.001

**Table 3:** Comparison of SAS and SDS score of two groups.

	Control group	Experimental group	*P* value
Self-rating anxiety scale			
Preoperation	55.3 ± 4.7	55.1 ± 4.3	0.891
3 weeks	40.0 ± 5.0	32.2 ± 5.8	<0.001

Self-rating depression scale			
Preoperation	56.1 ± 3.6	57.3 ± 3.9	0.123
3 weeks	40.0 ± 6.2	35.3 ± 4.8	<0.001

## Data Availability

All data included in this study are available upon request by contact with the corresponding author.

## References

[1] Plesh O., Wolfe F., Lane N. J. (1996). The relationship between fibromyalgia and temporomandibular disorders: prevalence and symptom severity. *Journal of Rheumatology*.

[2] Warren M. P., Fried J. L. J. C. T. O. (2001). Temporomandibular disorders and hormones in women. *Cells Tissues Organs*.

[3] LeResche M. L. J. C. R. O. B. (1997). Epidemiology of temporomandibular disorders: implications for the investigation of etiologic factors. *Critical Reviews in Oral Biology & Medicine*.

[4] Dworkin S. F., Huggins K. H., LeResche L. (1990). Epidemiology of signs and symptoms in temporomandibular disorders: clinical signs in cases and controls. *The Journal of the American Dental Association*.

[5] Katzberg R. W., Westesson D. P.-L., Tallents R., Drake C. M. J. J. O. M. S. (1996). Anatomic disorders of the temporomandibular joint disc in asymptomatic subjects. *Journal of Oral and Maxillofacial Surgery*.

[6] Fassicollo C. E., Machado B., Garcia D. M., Investigations C. D. F. J. C. O. (2019). Swallowing Changes Related to Chronic Temporomandibular Disorders. *Clinical oral investigations*.

[7] Yap A., Dworkin S. F., Chua E. K., List T., Tan K. B., Tan H. H. (2003). *Journal of Orofacial Pain*.

[8] Radwin L. E., Alster K. J. I. N. R. (2002). Individualized nursing care: an empirically generated definition. *International Nursing Review*.

[9] Suhonen R., Schmidt L. A., LJJoAN R. (2010). Measuring individualized nursing care: assessment of reliability and validity of three scales. *Journal of Advanced Nursing*.

[10] Mock V., Dow K. H., Meares C. J. (1997). Effects of exercise on fatigue, physical functioning, and emotional distress during radiation therapy for breast cancer. *Oncology Nursing Forum*.

[11] Lauver D. R., Ward S. E., Heidrich S. M. (2002). Patient-centered interventions. *Research in Nursing & Health*.

[12] Morgan S., Yoder L. H. J. JoH. N. (2012). A concept analysis of person-centered care. *Journal of Holistic Nursing*.

[13] Berg A., Hansson U. W., Hallberg I. R. J. JoA. N. (2010). Nurses’ creativity, tedium and burnout during 1 year of clinical supervision and implementation of individually planned nursing care: comparisons between a ward for severely demented patients and a similar control ward. *Journal of Advanced Nursing*.

[14] Sakurai M., Funashima N., mjjorfne Y. (2008). Individualized Nursing Care. *A Qualitative Study on Nursing Practice*.

[15] Kousoulou M., Suhonen R., Ajejoon C. (2019). Associations of individualized nursing care and quality oncology nursing care in patients diagnosed with cancer. *European Journal of Oncology Nursing*.

[16] Geng Y. Y., Wang B. J. C. JoC. (2020). Effect Observation of Individualized Nursing Intervention in Patients with Myocardial Infarction and Constipation.

[17] Charchalis M., Cossette S., Frasure-Smith N., Martorella G., Verville A., M-CGJCJo C. (2011). NP015 Development and Evaluation of an Individualized Nursing Intervention to Increase the Acceptance of Implantable Cardiac Defibrillators by New Carriers of These Devices. *Canadian Journal of Cardiology*.

[18] Huang X. J. A. (2021). Individual nursing promotes rehabilitation of patients with acute myocardial infarction complicated with arrhythmia. *American Journal of Tourism Research*.

[19] Małgorzata K., Małgorzata P., Kinga S., SJIjoer J., health p. (2021). Temporomandibular joint and cervical spine mobility assessment in the prevention of temporomandibular disorders in children with osteogenesis imperfecta. *A Pilot Study*.

[20] Garcia E., Flores R., Doherty J. J. O.N. A. (2022). Temporomandibular Joint Syndrome from an Ear versus Dental-Related Standpoint. *Otolaryngologic Clinics of North America*.

[21] Tanenbaum D., MJOcoNA L. (2022). Masticatory/temporomandibular disorders: practical assessment and care concepts for the otolaryngologist. *Otolaryngologic Clinics of North America*.

[22] Aroca J., Cardoso P., Favarão J. (2022). Auricular acupuncture in TMD-a sham-controlled, randomized, clinical trial. *Complementary Therapies in Clinical Practice*.

[23] Cintra D., de Oliveira S., Lorenzo I., Costa D., Bonjardim L., Costa Y. J. J. (2022). Detrimental Impact of Temporomandibular Disorders (Mis)beliefs and Possible Strategies to Overcome. *Journal of Oral Rehabilitation*.

[24] Tran C., Ghahreman K., Huppa C., Gallagher J. J. I., surgery M. (2022). Management of temporomandibular disorders: a rapid review of systematic reviews and guidelines. *International Journal of Oral and Maxillofacial Surgery*.

[25] Cândido Dos Reis A., Theodoro De Oliveira T., Vidal C., Borsatto M. (2021). Effect of auricular acupuncture on the reduction of symptoms related to sleep disorders, anxiety and temporomandibular disorder (TMD). *Alternative Therapies in Health and Medicine*.

[26] Peixoto K., da Silva Bezerra A., Melo R., de Resende C., de Almeida E., Barbosa B. (2021). Short-term effect of scalp acupuncture on pain, sleep disorders, and quality of life in patients with temporomandibular disorders: a A randomized clinical trial. *Pain Medicine*.

[27] Wang J., Zhou D., Dai Z., Li X. J. C. (2021). Association between systemic immune-inflammation index and diabetic depression. *Clinical Interventions in Aging*.

[28] Renton T., Beke B., pain f (2022). A narrative review of therapeutic peripheral nerve blocks for chronic orofacial pain conditions. *Journal of Oral & Facial Pain and Headache*.

[29] Rodhen R., de Holanda T., Barbon F., de Oliveira da Rosa W., Boscato B. (2022). Invasive surgical procedures for the management of internal derangement of the temporomandibular joint: a systematic review and meta-analysis regarding the effects on pain and jaw mobility. *Clinical Oral Investigations*.

[30] de Sire A., Marotta N., Ferrillo M. (2022). Oxygen-ozone therapy for reducing pro-inflammatory cytokines serum levels in musculoskeletal and temporomandibular disorders. *A Comprehensive Review*.

[31] Abreu Filho A., Tardivo L., Oliveira A., Silva H. J. A.-p. (2019). Brazilian Nursing and Psychology students’ visits to patients with amyotrophic lateral sclerosis: prospective analysis. *Arquivos de Neuro-Psiquiatria*.

[32] Cruz D., Monteiro F., Paço M. (2022). Genetic overlap between temporomandibular disorders and primary headaches: a systematic review. *Japanese Dental Science Review*.

